# Application of Deep Learning Model in Building Energy Consumption Prediction

**DOI:** 10.1155/2022/4835259

**Published:** 2022-08-08

**Authors:** Yiqiong Wang

**Affiliations:** School of Architectural Engineering, Sanmenxia Vocational and Technical College, Sanmenxia, Henan, China

## Abstract

In order to achieve China's energy conservation and emission reduction goal of peaking carbon dioxide emissions around 2030, it is of great significance. An important means of building energy conservation and emission reduction is the fine management of building energy consumption, which is based on the accurate prediction of building energy consumption, so as to support the optimal management of building operation and achieve the goal of energy conservation and emission reduction. This paper puts forward the evaluation indexes of the results of the building energy consumption prediction model, uses MAPE and RMSE indexes to evaluate the accuracy of the prediction results of the model, and uses the prediction time and input parameter dimensions to evaluate the time cost of the prediction model. Then, using the three building energy consumption prediction models based on machine learning algorithm established above, the prediction of energy consumption of four types of public buildings in different seasons is completed, and the prediction results are evaluated and analyzed. According to the prediction results and the requirements of related work on the accuracy of building energy consumption prediction model, the adaptation relationship between different types of buildings and different machine learning algorithm prediction models is summarized.

## 1. Introduction

In recent years, with the rapid development of human life, electricity consumption has also increased rapidly. Although solar energy, tidal energy, nuclear energy, wind energy, hydropower, and other clean and renewable energy sources have been widely used, today, fossil energy is still the main driving force for the development of human life as shown in Figure 1 [1]. The use of a large amount of fossil energy is undoubtedly accompanied by a large amount of greenhouse gas emissions. This has led to a rapid acceleration in global warming. As a major domestic power, China aims to achieve carbon dioxide emissions by 2030 to meet the common challenges facing all mankind. To achieve this goal, all aspects of Chinese life must make concerted efforts to promote energy conservation and emission reduction. As the economic foundation of the national economy, the construction industry not only promotes the development of relations, but also consumes a lot of energy [2]. According to statistics, in 2016, my country's electricity consumption reached 899 million tons of coal, accounting for 21% of the country's electricity consumption, of which 346 million tons were used for public housing models, accounting for 39% of the total construction. Therefore, promoting energy conservation and emission reduction in the construction industry is of great significance for reducing carbon dioxide emissions and achieving my country's 2030 carbon emission reduction goals as soon as possible. In the past energy-saving practices, various measures have been effectively utilized, and effective energy-saving effects have been achieved. In order to achieve the goal of building energy conservation and emission reduction, more regulation of energy efficiency is required [3]. Good household energy consumption management is an important part of future energy conservation development. The basis for this work is the massive building energy consumption data obtained through the energy consumption monitoring platform in recent years. The analysis and processing of domestic energy data can provide an important basis for the development of energy-saving technologies and the construction of energy-saving goals, the decomposition and utilization of water-saving materials and electric energy, and energy-saving testing. Although the national home appliance monitoring platform has been running for many years and has received many applications for home appliances, mining applications, and electronic data use, the house is not the breadth and depth it is now. On the other hand, this is due to the problems of missing values and variable costs in the home appliance data itself, resulting in insufficient data and unusable home appliances [4]. It has become possible to use the historical data of utility companies to predict the future of utility companies by developing predictive models through various machine learning algorithms. Because of the wide variety of buildings and jobs, there is no universal model to guide managers in choosing the approximate educational standards appropriate for different buildings, creating difficulties for leaders in appliance design. So, while many scientists have commented on the effectiveness of electronic estimates in certain buildings, there are questions about what machine algorithms are used in different households to achieve better home energy efficiency, and how global energy efficiency can be used. The technology to discuss the issues requires more research [5].

## 2. Related Works

Estimates for power plants began in the 1970s. Due to heat stress, people are thinking about controlling electricity consumption in households. At this time, Chen et al. began to use simple methods to calculate home energy efficiency [6]. Simple calculation methods solve the problem of constructing electrical estimation means from scratch, but they have shortcomings in estimation accuracy. To solve this problem, in the mid-1980s, Zhong et al. began to use statistical techniques to estimate building energy consumption and achieved good results [7]. With the continuous advancement of computer science and technology, Qin et al. began to try to use machine learning algorithms to predict household energy consumption in the 1990s [8]. After entering the new century, Goyal and Pandey do not like to limit by calculating capital. As the basis for machine learning algorithms, they started using cloud computing to speed up the process of building electronic simulations not only increasing the speed of computation, but also achieving more estimates of technical outcomes [9]. After decades of development, the prediction of building energy consumption has made remarkable progress. So far, the most widely used building energy consumption forecasting methods mainly include engineering simplification forecasting methods, physical model forecasting methods, and machine learning forecasting methods. Process technology is a technology that utilizes power generation technologies that have been described by many engineering disciplines. This method can be used to guide design work, estimating the initial stages of construction design. They are also widely used in practice due to the simplicity of engineering simplification forecasting methods. The physical prediction model uses the physical and electrical characteristics of the building to simulate the energy consumption process in the construction work through simulation software, so as to develop the thermal structure of the building, and achieves strong energy consumption and food estimates. Chen et al. found that the most commonly used physical model software is EnergyPlus, TRNSYS, DeST, and so on. [10]. Liu et al. found that when using the concepts of physics to create the best working model in the house, the physical estimation model needs to permeate many negative buildings, the environment is not good, and the design time is long [11]. At the same time, because the construction is not good, the environment is no different from different buildings in the actual project, and each house has to redesign the structure to estimate the energy, so this method is difficult to repeat. Machine learning prediction methods are data-driven models that can estimate power consumption from historical data mining. This approach eliminates the disadvantage of a large number of parameter inputs in physical modeling. Once the algorithm model is established, the energy consumption of the building can be simulated and predicted based on historical data, which undoubtedly greatly increases the repeatability of the model. It also supports the research and improvement of applications based on machine learning algorithms. According to international standards, many scientists have refined the process according to the characteristics of home appliances to meet the needs of research. Wei and Isler through the impact study [12] applied the data mining system to the operation of domestic air conditioners in line with international standards. Chen et al. linked power consumption estimation with user behavior analysis to provide a new data mining process after considering the form of home air conditioning system and the actual usage behavior of users [13]. In order to achieve the purpose of home appliances and diagnose problems, Sun et al. combine the influence of home appliances and electricity consumption, and the workflow of applying data mining includes four stages of data distribution and conversion, data analysis, data mining, and data mining [14]. The Hong Kong Polytechnic University research team compiled a data mining workflow including data preprocessing, grouping analysis, correlation analysis, and postprocessing based on the Hong Kong International Financial Center building automation system data and existing performance laboratory research—machining and application knowledge to understand the benefits of improved diagnostics. As can be seen from the research and analysis of impact studies, only three main tasks are required for household electronics usage data: data selection and processing, design and assembly, and testing and implementation [15]. Power plants estimated using the data as part of data mining do not yet have significant operational procedures.

## 3. Method

As shown in Figure 2, McCulloch and Pitts jointly proposed the basic processing unit of artificial neural networks: M-P neuron model.

*x*_1_, *x*_2_, *x*_3_,…, *x*_*n*_ is the input of neurons, *w*_1_, *w*_2_, *w*_3_,…, *w*_*n*_ is the input intensity of stimulating neurons, *θ* is the threshold, and the output is ∑_*k*=1_^*n*^*x*^*k*^*w*^*k*^ − *θ*, where Σ is the accumulator. Only when the output is greater than 0, the neuron is activated; otherwise, it is in an inhibitory state [16]. *F* is the activation function. When *y* is used to represent the final output of neurons, the signal processing process can be expressed by

(1) $$\begin{array}{c} y=f\left(\sum_{k=1}^{n}x^{k}w^{k}-\theta \right). \end{array}$$

If the threshold *θ* is regarded as a weight *w*_0_ of specific input *x*_0_, formula (1) can be simplified to

(2) $$\begin{array}{c} y=f\left(\sum_{k=0}^{n}x^{k}w^{k}\right). \end{array}$$

The perceptron proposed by Frank Rosenblatt is a linear binary classification model based on the “M-P” model: input the feature vector of *n*-dimensional real number. After linear combination, when the result is greater than a certain number, output is 1, otherwise output −1. It can be expressed by

(3) $$\begin{array}{c} f\left(x_{0},x_{1},x_{2},x_{3},\ldots ,x_{n}\right)=\left\{\begin{array}{cc} 1, & \sum_{k=0}^{n}x_{k}w_{k}\geq 0,\\ -1, & \sum_{k=0}^{n}x_{k}w_{k}\leq 0. \end{array}\right) \end{array}$$

Frank Rosenblatt gave the proof that the algorithm must converge when the two types of modes are linearly separable (i.e., there is a hyperplane to separate the two types of modes) [17].  Table 1 takes a single-layer perceptron with two inputs as an example (the threshold value is to shift the linear value and ignore the threshold value temporarily), showing the relationship between AND, OR, NOT, and XOR.

Logical AND, OR, NOT (*x*1), and NOT (*x*2) can all use a straight line to separate the results 0 (false) and 1 (true). However, due to the limitations of single-layer perceptron, XOR cannot be classified; that is, the problem of nonlinear segmentation cannot be solved. The logic XOR is shown in Figure 3.

Many linear inseparable problems can realize the segmentation of complex space through multiple layers and multiple perceptrons. The two linear classifiers of the first layer perceptron divide the feature space into two parts and then use the linear combination as the input of the second layer perceptron, so as to realize the spatial segmentation of XOR operation:

(4) $$\begin{array}{c} y=\theta \left\{\sum_{j=1}^{n}v_{j}\theta \left(\sum_{i=1}^{m}w_{ij}x_{i}+w_{oj}\right)+v_{o}\right\}, \end{array}$$

where *θ*(·) in equation (4) is a step function. Kolmogorov's theory points out that the double hidden layer perceptron can solve any complex classification problem [18]. However, the complexity of practical problems is more complex than XOR problems, so it is necessary to build a multi-layer network to solve complex problems. Such a multi-layer structure is called neural network, and the model trained by multi-layer neural network is called deep learning model. Formula (1) shows the function of activation function, and different activation functions will make the neural network have different characteristics. Several commonly used activation functions are described below: ladder function formula (5), sigmoid function formula (6), tanh hyperbolic function formula (8), and ReLU modified linear unit function formula (10). Ladder function is relatively simple and generally used for teaching. The formula is as follows:

(5) $$\begin{array}{c} \text{Step function such as}\left(5\right):f\left(x\right)=\left\{\begin{array}{cc} 1, & x>0,\\ 0, & x\leq 0, \end{array}\right) \end{array}$$

(6) $$\begin{array}{c} \text{Sigmoid function}:f\left(x\right)=\frac{1}{1+e^{-x}}. \end{array}$$

As shown in Figure 4, sigmoid is a continuous and differentiable function everywhere. It has very good nonlinear characteristics. Therefore, when it is applied to multiple different neurons, the output result is also nonlinear.

Formula (7) is the derivative of sigmoid:

(7) $$\begin{array}{c} f\left(x\right)=\frac{e^{-x}}{{\left(1+e^{-x}\right)}^{2}}\\ =\left(\frac{1}{1+e^{-x}}\right)\left(1-\frac{1}{1+e^{-x}}\right)\\ =f\left(x\right)\left(1-f\left(x\right)\right). \end{array}$$

Figure 5 shows the derivative function image of sigmoid. When the value of *X* is around the value of 0, the derivative value is large, which means that small changes in independent variables can cause large changes in dependent variables. Therefore, it is very suitable to divide the output value of dependent variables into different value ranges, which will have a better signal feature space mapping effect. In Figure 5, the value change of the area where the sigmoid derivative falls outside [−3, 3] is very small and gentle, and when the derivative result falls into this area, the value is close to 0, resulting in the disappearance of the gradient [19]. The value range of sigmoid function is (0, 1), so the input of the next neuron is limited to the (*o*, 1) interval, which is a very obvious limitation of sigmoid.

(8) $$\begin{array}{c} \text{Hyperbolic function}:f\left(x\right)=\frac{e^{2x}-1}{e^{2x}+1}. \end{array}$$

As shown in Figure 6, the value range of hyperbolic function is (−1, 1) and is completely symmetrical, so it makes up for the deficiency that the value range of sigmoid function is only positive, but other characteristics are very similar to sigmoid function. Hyperbolic functions are continuously differentiable in the domain of definition.

(9) $$\begin{array}{c} \text{Hyperbolic derivative}:f\left(x\right)=1-{\left(\frac{e^{2x}-1}{e^{2x}+1}\right)}^{2}. \end{array}$$

Whether sigmoid or tanh is selected depends on the gradient requirements in practical problems. Similar to sigmoid, tanh also has gradient disappearance.  Figure 7 shows that the tanh gradient outside a certain value area is very small.

Tom Michael Mitchel explained the concept of machine learning in his book machine learning: assuming that the computer's performance measured by P for a certain task *t* can be improved from me based on experience *E*, it is said that the computer program can learn from experience *E*. Traditional machine learning requires manual extraction of parameters that affect the classification results, but deep neural network (deep neural network with hidden layer greater than 2) can learn various features of entities by itself and combine simple features into more complex and more abstract features, so as to use these combined abstract features to solve the problem. Therefore, deep learning has made a breakthrough in traditional machine learning to some extent, which has promoted the prosperity and development of artificial intelligence in many fields. For example, the image recognition based on winder neural network has achieved quite high prediction accuracy, the natural language processing system based on long-term and short-term memory network has also made great progress, and the deep learning based on multi-layer general regression neural network has also achieved many results, such as the prediction of thermal effect of solar air heater [20, 21].

In addition, the energy consumption prediction model is proposed to explain the reasons for the model performance degradation, and the law of model error is mined to construct a faster and more comprehensive prediction model logic. It provides ideas for model reliability evaluation and is conducive to improving the practical value of complex data-driven models in building energy consumption prediction applications.

First, the sensitivity index of the model input is calculated based on the sensitivity analysis method, which is used to measure the influence of the model input on the predicted value of energy consumption; then, the weighted Manhattan distance between the predicted condition and the training set is calculated based on the sensitivity index, which is used to quantify the predicted condition. Finally, based on the error and distance data, the relationship between the prediction error and the weighted Manhattan distance is fitted, which is used to infer the variation law of the model prediction error and evaluate the reliability of the model. The traditional data-driven energy consumption prediction model has high complexity, the prediction process is a black box, and the interpretability is poor. Sensitivity analysis is suitable for analyzing the influence of independent variable changes on the target result, which can effectively quantify the influence of each input feature on the predicted value of energy consumption, thus reflecting the response of the prediction model to the input feature. Sensitivity analysis has been widely used in areas such as supply chain management, sustainable energy production, and industrial manufacturing.

Building energy consumption prediction is the basis for subsequent optimal operation, fault detection, and energy-saving evaluation. Information such as the potential error variation law and reliability of the prediction model is of great significance for relevant energy system management decisions. Based on the weighted Manhattan distance and the model prediction error data of the prediction conditions and the training set, the relationship between the two can be further explored, the variation trend of the model prediction error with the weighted Manhattan distance can be revealed, and the extrapolation ability and reliability of the model in the face of unknown conditions can be analyzed. It can provide more comprehensive information for the subsequent optimization operation, fault detection, and diagnosis based on the prediction results. The linear regression method has a simple principle and strong interpretability, and is suitable for fitting the relationship between the model prediction error and the weighted Manhattan distance. First, take the logarithm of the prediction error and the weighted Manhattan distance to reduce the heteroscedasticity; then define the relationship between the positive error and the negative error and the distance, as shown in (10) and (11); then use the least squares method to fit undetermined parameters *a*1, *b*1, *a*2, and *b*2 in the relational expression; finally, according to the statistical distribution of errors, move the fitting curve up and down as the upper and lower boundaries of the error interval, until the number of error points in the interval meets the given confidence level. Then, the two boundary lines form the confidence interval for the forecast error.

(10) $$\begin{array}{c} {\text{log}}_{10}\left(e_{p}\right)=a_{1}{\text{log}}_{10}\left(D\right)+b_{1},e_{p}>0, \end{array}$$

(11) $$\begin{array}{c} -{\text{log}}_{10}\left(\left|e_{n}\right|\right)=a_{2}{\text{log}}_{10}\left(D\right)+b_{2},e_{p}<0, \end{array}$$

where *D* is the weighted Manhattan distance between the prediction condition and the training condition, *e*_*p*_ is the positive prediction error of the model, *e*_*n*_ is the negative prediction error of the model, and *a*_1_, *b*_1_, *a*_2_, and *b*_2_ are undetermined parameters. According to the fitting relationship between error and distance, the variation law of prediction error with distance can be obtained, which can be used to explain when the prediction model has large error and low reliability. Faced with the unknown working conditions to be predicted, the prediction error of the model can be inferred according to the relationship. If the error exceeds the given threshold, it means that the performance of the prediction model is attenuated greatly and the reliability is low, and needs to be corrected.

## 4. Experiment and Analysis

With the popularity of data-driven models in various fields, their interpretability has also received more and more attention. The complex structure of machine learning models or deep learning models enables them to learn complex relationships between building energy consumption and related variables, but it also makes the relationships and prediction processes they learn difficult to explain with human knowledge. There have been a lot of studies on the application of data-driven models in the field of building energy consumption prediction, but there are few studies on the interpretation methods of data-driven models. A general explanation process for energy consumption prediction models is proposed, which can explain the influence of model input on the predicted value, mine the variation law of model error, and evaluate the reliability of the model.

The training process includes the setting and comparison test of various super-parameters. The super-parameters involved in the adjustment include depth of neural network, number of nodes in hidden layer, activation function, learning rate, attenuation coefficient, regularity coefficient, etc. Through the continuous adjustment and optimization of various super-parameters, the training results of different parameter combinations are analyzed and compared, and the better parameter combination is selected [22, 23]. When the detailed meteorological data are used as the input data, the input layer will have 91059-dimensional data. When the first hidden layer uses more than 91059-dimensional nodes, the computer memory usage exceeds 32 GB, and the memory will overflow. If the first hidden layer uses fewer nodes, it can only continue to increase the number of hidden layers. When it is increased to 7 hidden layers, it is very difficult to adjust the optimization parameters. Due to the limitation of hardware environment, this paper uses climate region vector instead of meteorological data as training input and obtains good results [24]. The brief introduction of the development platform environment is shown in Table 2.

The normalized data are a CSV file. Each row of data contains the scalar of energy consumption parameters affecting the building and the corresponding EUI energy consumption data. These data need to be processed and divided again in order to really input the deep learning model for training. The randomly divided data set is divided into four files [25, 26], as shown in Table 3.

The EUI value distribution of training data is shown in Figure 8.

To sum up, we can see that the climate regional distribution and EUI distribution of training data set, validation data set, and real-time test data set are very similar. This can ensure the consistency between training and verification. That is, all situations are trained during training and verified during verification, which greatly improves accuracy of results. The accuracy evaluation measure of classification problem is accuracy, but the regression problem is not suitable for this method. Therefore, this paper uses the evaluation measure for predicting continuous values, which is divided into quantitative and qualitative evaluation methods. The evaluation benchmark data of experimental results are the EUI output of DOE-2 simulation calculation engine. This paper not only compares the results of deep learning models based on different parameters, but also compares the results of deep learning models with those of other machine learning models. Finally, it also makes a horizontal comparison and analysis with similar problems of other scholars. Sigmoid as a neuron activation function model has achieved a relatively good prediction value. It can be seen that more than 83% of the verification building error is within 20%. The parameters of the model with ReLU as the activation function are more difficult to adjust, which is related to the characteristics of unilateral inhibition of ReLU. After neuron calculation, it can only output positive value, so the neuron pruning force using ReLU is greater, and it is more difficult to predict the specific values in this paper.

The prediction error of tanh as the activation function model is also large. The analysis shows that it may be related to the normalization method of training data. The normalization method used in this paper makes all data fall in the range of [0, 1], but the numerical sensitivity interval of tanh activation function is more appropriate between [−1, 1]. The deep learning model with sigmoid as the activation function takes the best prediction result in the deep learning model. The experimental results also show that it is feasible to use deep learning to predict building energy consumption, and can achieve high accuracy [27].

Specifically, the sensitivity indices (*I*) of 96 input variables of the three mixed models LSTM-BPNN, CIFG-BPNN, and GRU-BPNN were calculated to reveal the influence of different input variables on the load prediction value. After data normalization, all input variables have been normalized to [0, 1], so the input variable reference value is 0.5, the variation range of each input variable is from 0.25((100% − 5 × 10%) × 0.5) to 0.75 ((100% + 5 × 10%) × 0.5), and the step size is 0.05; that is, 1 takes 5, and △ takes 10%.

The sensitivity index (*I*) of each variable in different cases, comparing the sensitivity index of different variables, can be found that the impact of historical cooling load on the model output far exceeds other variables. Similar conclusions were also found by comparing the prediction accuracy of the models when using different input features. The historical cooling load has a great influence on the predicted value of the future cooling load, and the influence of the historical load closer to the prediction time is greater. The result is consistent with the actual load variation rule under the influence of the thermal inertia of the building, which indicates that the hybrid model is used for feature extraction. The thermal inertia can be taken into account when considering the thermal inertia, focusing on the input characteristics related to thermal inertia; the cooling load 24 hours ago and 23 hours ago also has a certain impact on the predicted value; this is because the cooling load change cycle is about 24 hours, the same time every day. The cooling loads are similar, indicating that the hybrid model captures the periodicity of building operation.

In order to verify the validity of the general interpretation process of the energy consumption prediction model, this process is used to explain the hybrid model and the comparison model. Using building cooling load data and experimental cases, the experimental results show (1) that the historical cooling load has the greatest impact on the predicted value, the time variable (hours) and outdoor temperature also have a certain impact on the predicted value, and the effect of outdoor relative humidity is very small; (2) that the weighted Manhattan distance of the test case in 2 is significantly larger than the weighted Manhattan distance of the test case in case 1, so the same prediction model will produce a large performance degradation in the case; and (3) the logarithm of the model prediction error and the weighted Manhattan distance pair. The number is basically linear. The larger the distance, the larger the model prediction error and the more inaccurate the model. In practical applications, the distance can be used to determine whether the model prediction result is reliable. The above conclusions show that the proposed energy consumption prediction model interpretation process can quantify the influence of model input on the predicted value, explain the reasons for the decline of model performance, and discover the variation law of model errors, which improves the interpretability and reliability of data-driven models. Building energy management provides reliable decision support.

## 5. Conclusion

With the rise of green homes, more and more attention has been paid to the analysis of appliances through the use of software development during the design phase. More and more simulation software will be used for the design and reconstruction of buildings, and then the actual energy consumption will be higher and higher. For the rapid analysis of the design simulation software and the rapid feedback given according to the selection, this paper proposes to use deep learning to predict the building energy consumption and use the existing building energy consumption data for training. In the building energy consumption prediction task of deep learning, the processing schemes of various building parameters are proposed, so that the deep learning model can use these parameters, create a deep learning model suitable for this task, and use a variety of optimization algorithms of deep learning to optimize various parameters. Firstly, it introduces the environment and development platform used in the experiment, as well as the training and prediction of the data set used. Then, it explains the evaluation methods used in this experiment, mainly using root mean square error (RMSE) and average absolute percentage error (MAPE) as quantitative evaluation, and compares the prediction results of validation data sets on different models. The determination coefficient (*R*2) is used as a qualitative evaluation to explain the prediction correlation and prediction ability of the prediction model. By comparing the prediction results of deep learning model, multiple linear regression, support vector regression model, and common machine learning models of other scholars, the deep learning model using sigmoid as activation function has achieved better prediction results, which proves that deep learning is feasible in building energy consumption prediction to a certain extent. In order to improve the application reliability of data-driven models, a general explanation process for energy consumption prediction models is proposed, which quantifies the impact of input on predicted values, explains the reasons for model performance degradation, and explores the variation law of model prediction errors, providing ideas for model reliability assessment. The experimental results show that the method can explain and analyze the prediction model from many aspects, and realize the quantitative evaluation of the reliability of the model. The application of the general interpretation process of energy consumption prediction models in practical projects can improve the interpretability and application reliability of data-driven models, and promote the further promotion and application of data-driven models in buildings and other fields.

## Figures and Tables

**Figure 1:** Smart building with zero energy consumption.

**Figure 2:** M-P neuron model.

**Figure 3:** Logic XOR.

**Figure 4:** Sigmoid function.

**Figure 5:** Sigmoid derivative.

**Figure 6:** Hyperbolic function.

**Figure 7:** Derivative of hyperbolic function.

**Figure 8:** EUI distribution of training data.

**Table 1:** Boolean algebraic representation of single-layer perceptron.

*X*_1_	*X*_2_	AND	OR	NOT (*x*_1_)	NOT (*x*_2_)	XOR
0	0	0	1	1	1	0
0	1	0	1	1	0	1
1	0	0	0	0	1	1
1	1	1	0	0	0	0

**Table 2:** Introduction to development platform.

Serial number	Platform usage tools	Version information
1	Development language	Python2.7
2	Scientific computing tool library	NumPy, scikit-learn
3	Computational framework	TensorFlowl.6
4	Data extraction and storage	MongoDB3.2

**Table 3:** Overview of data sets.

Data set file	Content of each line	Purpose	Data row	Remarks
Training set	Building parameters 3461 dimensions	Train	33116	Last dimension: EUI Penultimate two-dimensional: meteorological data key value
Validation set	Building parameters 3461 dimensions	Verification	2070	Last dimension: EUI Penultimate two-dimensional: meteorological data key value
Real-time test set	Building parameters 3461 dimensions	Real-time test	202	Last dimension: EUI Penultimate two-dimensional: meteorological data key value
Climate set (some)	Climate data 87600 dimensions	Supplementary training set	1	Supplement the first three data sets

## Data Availability

The data underlying the results presented in the study are available within the article.
